# Suppression of AP1 Transcription Factor Function in Keratinocyte Suppresses Differentiation

**DOI:** 10.1371/journal.pone.0036941

**Published:** 2012-05-23

**Authors:** Bingshe Han, Ellen A. Rorke, Gautam Adhikary, Yap Ching Chew, Wen Xu, Richard L. Eckert

**Affiliations:** 1 Department of Biochemistry and Molecular Biology, University of Maryland School of Medicine, Baltimore, Maryland, United States of America; 2 Department of Dermatology, University of Maryland School of Medicine, Baltimore, Maryland, United States of America; 3 Department of Obstetrics, Gynecology and Reproductive Sciences, University of Maryland School of Medicine, Baltimore, Maryland, United States of America; University of Tennessee, United States of America

## Abstract

Our previous study shows that inhibiting activator protein one (AP1) transcription factor function in murine epidermis, using dominant-negative c-jun (TAM67), increases cell proliferation and delays differentiation. To understand the mechanism of action, we compare TAM67 impact in mouse epidermis and in cultured normal human keratinocytes. We show that TAM67 localizes in the nucleus where it forms TAM67 homodimers that competitively interact with AP1 transcription factor DNA binding sites to reduce endogenous jun and fos factor binding. Involucrin is a marker of keratinocyte differentiation that is expressed in the suprabasal epidermis and this expression requires AP1 factor interaction at the AP1-5 site in the promoter. TAM67 interacts competitively at this site to reduce involucrin expression. TAM67 also reduces endogenous c-jun, junB and junD mRNA and protein level. Studies with c-jun promoter suggest that this is due to reduced transcription of the c-jun gene. We propose that TAM67 suppresses keratinocyte differentiation by interfering with endogenous AP1 factor binding to regulator elements in differentiation-associated target genes, and by reducing endogenous c-jun factor expression.

## Introduction

Activator protein one (AP1) transcription factors are a family of jun and fos proteins that form jun-jun and jun-fos homo- and heterodimers, and these complexes interact with AP1 factor DNA binding sites to regulate gene expression [1]–[4]. The AP1 factor family includes c-jun, junB, junD, c-fos, FosB, Fra-1 and Fra-2. These proteins are implicated in control of keratinocyte proliferation [5]–[7], differentiation [8]–[10], apoptosis [11], [12], and transformation [13]–[16]. The importance of these proteins is confirmed by in vivo studies [13], [17]–[25]. Analysis of the role of these proteins in epidermis is complicated because AP1 proteins display context-dependent functions and because multiple family members are expressed.

An altered form of c-jun, which is truncated to remove the N-terminal transactivation domain, has been used to study AP1 factor function [26]. Deletion of the c-jun transactivation domain creates a dominant-negative form of the protein (TAM67) that inhibits AP1 factor function [26]. TAM67 has been used in a number of systems. TAM67 expression in lung cancer in mice [27], [28] and in nasopharyngeal carcinoma inhibits cell growth by altering cell cycle protein expression [29]. TAM67 inhibits growth of MCF-7 breast cancer cells [30], and halts HT-1080 cell proliferation in G1 phase [31]. TAM67 has also been used to study the impact of AP1 factor signaling on cell differentiation. Inhibition of AP1 factor function in neuroblastoma cells suppresses nerve growth factor-dependent differentiation [32]. In melanoma cells, induction of the melanoma differentiation associated genes is increased by AP1 factors and inhibited by TAM67 [33], and TAM67 also inhibits differentiation in monocytic leukemia cells [34].

We [35], [36] and others [37]–[43] have used TAM67 to study AP1 factor function in keratinocytes. These studies show that TAM67 inhibits keratinocyte differentiation [35], [36]. Cell culture based studies in human primary foreskin keratinocytes show that AP1 factors are required for expression of markers of terminal differentiation and that inhibition of AP1 factor function with TAM67 suppresses these responses [10], [36], [44]. We have also recently shown that expression of TAM67 in vivo in suprabasal mouse epidermis results in delayed and incomplete epidermal differentiation [35].

However, the molecular mechanism of TAM67 action in these models is not fully understood. In the present study we examine the mechanism of TAM67 action on AP1 factor function in epidermal keratinocytes. These studies indicate that TAM67 homodimer binds to AP1 factor DNA binding sites in human keratinocytes to inhibit jun and fos factor binding, and also reduces the mRNA and protein level of endogenous jun family members. In the case of c-jun this is via inhibition of transcription. Moreover, TAM67 binding to the AP1-5 binding site of the involucrin (hINV) promoter reduces expression of involucrin, a keratinocyte differentiation marker, in cultured keratinocytes. We further show that TAM67 in murine epidermis reduces involucrin (and loricrin) gene expression and reduces binding of endogenous AP1 factors to AP1 factor binding elements.

## Results

TAM67 is a truncated form of c-jun that lacks the amino terminal transactivation domain and is not transcriptionally active [26] (**Fig. 1A**). In the present study we utilize TAM67 as a tool to study AP1 factor function in normal human keratinocytes. To initiate these studies, we monitored TAM67-FLAG expression. **Fig. 1B** shows that TAM67-FLAG is expressed in keratinocytes and **Fig. 1C** shows that, as expected of a nuclear transcriptional regulator, TAM67-FLAG accumulates in the nucleus.

**Figure 1:** TAM67-FLAG expression in keratinocytes. A Comparison of c-jun and TAM67 structure. The numbers are indicated in amino acids. The transactivation, DNA binding and leucine zipper domains are indicated. The TAM67 truncated protein is FLAG epitope tagged as indicated. **B/C** TAM67-FLAG is expressed in keratinocytes. Normal human keratinocytes were infected with 10 MOI of tAd5-EV or tAd5-TAM67-FLAG with 5 MOI of Ad5-TA. After 24 h the cells were fixed for immunostaining and extracts were prepared for immunoblot with anti-FLAG. Similar results were observed in each of three repeated experiments.

AP1 factors are key regulators of function in keratinocytes [45]–[47]. To understand the impact of TAM67 on AP1 factor function, we monitored endogenous AP1 factor level in TAM67-expressing cells. **Fig. 2A** shows a reduction in c-jun, junB and junD but no change in Fra-1, Fra-2 or c-fos level in TAM67 expressing cells, suggesting that TAM67 reduces the level of a subset of AP1 factors. To assess the mechanism causing c-jun, junB and junD reduction, we monitored mRNA level using quantitative RT-PCR. The level of c-jun, junB and junD encoding mRNA is reduced in TAM67 expressing cells, indicating that part of the reason for loss of these factors is a reduction in mRNA level (**Fig. 2B**). In contrast, the level of RNA encoding fos family members (Fra-1, Fra-2, c-fos) is not altered. We next examined the ability of TAM67-FLAG to interact with other AP1 factors by testing the ability of TAM67-FLAG to co-precipitate individual AP1 factors in keratinocytes. As shown in **Fig. 2C**, anti-FLAG precipitation of TAM67-FLAG co-precipitates Fra-1, Fra-2 and c-fos. In contrast, junB and junD did not co-precipitate, which is expected considering that these proteins are reduced in level in TAM67-expressing cells (**Fig. 2A**). In spite of the reduction in total c-jun level (**Fig. 2A**), sufficient c-jun appears to remain and interacts with TAM67-FLAG (**Fig. 2C**). We next monitored the impact on nuclear AP1 factor level. **Fig. 2D** shows that TAM67 expression is associated with reduced nuclear c-jun, junB and junD. In contrast, nuclear c-fos, Fra-1 and Fra-2 levels are not affected.

**Figure 2:** Impact of TAM67-FLAG on AP1 factors. Keratinocytes were infected with empty (EV) or TAM67-FLAG encoding adenovirus and after 24 h cells were harvested and extracts prepared. **A** Total extracts were electrophoresed for immunoblot detection of the indicated proteins. **B** TAM67-FLAG suppresses jun factor mRNA level. At 24 h post-infection with EV or TAM67-FLAG encoding virus, mRNA was prepared for detection by quantitative PCR. The bars are mean ± SD and the asterisks indicate a significant reduction (p<0.005, n = 3). **C** Total extract (200 µg) was immunoprecipitated with anti-FLAG and the immunoprecipitate was electrophoresed for immunoblot to detect the indicated jun and fos proteins. **D** Nuclear extract was prepared and the level of each indicated protein was measured by immunoblot. Similar results were observed in three experiments.

### TAM67-FLAG Impact on c-jun Gene Expression

As shown above, c-jun, junB and junD protein and mRNA levels are reduced in TAM67-expressing cells. To gain insight regarding the mechanism, we used c-jun as a model. We examined the impact of TAM67 on c-jun mRNA level and promoter activity in a side-by-side comparison. **Fig. 3A** shows that TAM67 reduces c-jun encoding mRNA by more than 50%. To gain insight into the mechanism, we monitored the impact of TAM67 on activity of a c-jun promoter construct in which nucleotides −1780/+731 is linked to luciferase (**Fig. 3B**). Our studies show that TAM67 reduces promoter activity by 50% in keratinocytes. In contrast, the same promoter in which the key AP1 factor binding sites are mutated, −1780/+731(AP1m) [48], displays basal activity and is not regulated by TAM67. **Fig. 3C** shows the structure of the promoter constructs. These findings suggest that c-jun level is reduced by a transcriptional mechanism that requires AP1 factor binding sites in the c-jun promoter upstream regulatory region.

**Figure 3:** TAM67 suppresses c-jun promoter activity. **A** TAM67 reduces c-jun mRNA. Keratinocytes were infected with empty (EV) or TAM67-FLAG encoding adenovirus (10 MOI) and after 24 h mRNA was prepared and c-jun mRNA level was measured by quantitative PCR. **B** TAM67 suppresses c-jun promoter activity. Keratinocytes were transfected with 1 µg of the indicated c-jun promoter luciferase reporter construct and 1 µg of pcDNA3 (EV) or pcDNA3-TAM67-FLAG (TAM67-FLAG). After 24 h the cells were harvested and assayed for luciferase activity. The values in both plots are mean + SD and the asterisks indicate a significant reduction (p<0.005, n = 3). **C** Map of c-jun promoter region. The promoter constructs encode nucleotides −1780 to +731 with the transcription start site at +1. c-jun(−1780/+731) is the wild-type intact promoter and c-jun(−1780/+731)-AP1m is a construct in which the critical AP1 sites are eliminated by mutation [48]. LUC indicates the luciferase gene. The numbers are given in nucleotides.

### TAM67-FLAG Inhibits AP1 Factor Binding to AP1 Consensus DNA Binding Element

Gel mobility shift and supershift analysis, using a consensus AP1 binding probe, was performed to investigate the effect of TAM67-FLAG on AP1 factor interaction with DNA. **Fig. 4A** shows a gel shift using ^32^P-labeled AP1 consensus binding site oligonucleotide and human foreskin keratinocyte nuclear extract. Shifted bands appear at increased intensity and free probe appears at reduced intensity in nuclear extracts prepared from TAM67-FLAG expressing cells (lanes 3, 5 and 9). This is caused by an increase in total cellular AP1 site binding capacity due to the presence of TAM67. As expected, addition of anti-FLAG results in appearance of a supershifted band only in extracts from TAM67-FLAG expressing cells (lane 5, asterisk). We next incubated nuclear extract from control and TAM67-expressing cells with anti-c-jun, junB, junD, Fra-1, Fra-2, c-fos or fosB. Supershifted bands are observed for each AP1 factor. The most obvious supershifts were observed for c-jun, junD, Fra-1, Fra-2 and c-fos (**Fig. 4B**). The amount of supershifted DNA is reduced in TAM67-expressing cells, demonstrating that TAM67 competes for endogenous AP1 factor binding to the AP1c element (**Fig. 4B**). We also examined the ability of TAM67 to form dimers. Nuclear extract from TAM67-FLAG expressing cells was crosslinked with disuccinimidyl suberate (DSS) prior to denaturing gel electrophoresis. **Fig. 4C** shows the presence of a TAM67 dimer, in DSS-treated extracts, migrating at 54 kDa. There are also higher molecular weight forms (brackets) which most likely represent TAM67 crosslinking to endogenous AP1 factors. However, the major band appears as a TAM67 homodimer. These findings suggest that TAM67 homodimers interact with AP1 binding sites to inhibit binding of endogenous AP1 factors. It also suggests that a TAM67 homodimer may be the major AP1 site interacting species in these cells.

**Figure 4:** TAM67-FLAG inhibits AP1 factor binding to AP1 consensus DNA binding element. Keratinocytes were infected with 10 MOI tAd5-EV or tAd5-TAM67-FLAG and after 24 h nuclear extracts were prepared. **A** AP1 factors interact with AP1 consensus DNA element. Nuclear extracts were incubated with AP1c-P^32^ without or with a 50-fold molar excess of Sp1c or AP1c oligonucleotides, or anti-FLAG antibody and electrophoresed on a 6% acrylamide non-denaturing gel. FP indicates free probe and NE is nuclear extract. The arrow indicates the major shifted band and asterisks indicate migration of supershifted complexes. AP1c and Sp1c encode consensus AP1 and Sp1 binding elements. **B** TAM67-FLAG reduces AP1 factor binding to DNA. Nuclear extracts were incubated with AP1c-P^32^ in the absence or presence of c-jun, junB, junD, Fra-1, Fra-2, c-fos, or fosB antibodies, and electrophoresed on a 6% acrylamide non-denaturing gel. Arrows indicate shifted band and asterisks supershifted bands. FP indicates free probe. **C** TAM67-FLAG forms homodimers and heterodimers. Nuclear extracts were treated with or without DSS crosslinker prior to electrophoresis on a denaturing 8% polyacrylamide gel and TAM67-FLAG was detected by anti-FLAG immunoblot. Identical results were observed in three repeated independent experiments.

### TAM67-FLAG Inhibits hINV Gene Expression

We next investigated the impact of TAM67 on AP1-regulated gene expression using involucrin (hINV) as an AP1 responsive gene [10]. Involucrin is a keratinocyte differentiation marker and is known to be increased by AP1 transcription factor signaling [25], [47], [49]–[51]. Control and TAM67-FLAG expressing keratinocytes were harvested and the level of hINV protein and mRNA was measured. **Fig. 5A** shows a TAM67-dependent reduction in hINV protein and mRNA. To assess the mechanism, we monitored the impact on hINV promoter activity. Three promoter constructs were used and keratinocytes were treated with TPA, a strong inducer of AP1-dependent hINV promoter activity [47], [49]. The hINV basal promoter, which encodes 41 nucleotides upstream of the transcription start site [47] and no AP1 sites, is not regulated by TAM67 or TPA (**Fig. 5B**). In contrast, pINV-241, which encodes the proximal regulatory region, and pINV-2473, which encodes both the proximal and distal regulatory regions [23], [47], are responsive to TPA and basal and TPA-stimulated promoter activity is inhibited by TAM67. The proximal and distal regulatory regions encode regulatory elements required for promoter activity in cultured keratinocytes [47] and involucrin expression *in vivo* [47], [49]. These experiments indicate that TAM67 inhibits differentiation-associated AP1-dependent transcriptional events in keratinocytes.

**Figure 5:** TAM67-FLAG inhibits hINV gene expression. **A** TAM67 reduces hINV protein and mRNA level. Keratinocytes were infected with indicated MOI of tAd5-EV or tAd5-TAM67-FLAG and after 48 h extracts were prepared to detect hINV protein by immunoblot and mRNA by quantitative PCR. The values are mean ± SD and the asterisks indicate a significant reduction using student’s t-test, n  = 3 (p<0.001). **B** TAM67 suppresses AP1 factor-dependent promoter activity. Keratinocytes were transfected with the indicated hINV reporter constructs in the presence of empty pcDNA3 vector or pcDNA3-TAM67-FLAG and treated 24 h with or without 50 ng/ml TPA prior to preparation of extracts and assay of luciferase activity. The values are mean ± SEM and the asterisks indicate a significant reduction using student’s t-test, n = 3 (p<0.001).

### TAM67-FLAG Binds to the AP1-5 Site of hINV Gene Promoter

AP1 factors regulate transcription of hINV via binding to the proximal and distal AP1 sites in the hINV promoter [25], [47], [49]–[51]. In particularly, the AP1-5 site in the distal promoter is absolutely required for involucrin gene expression *in vivo* [22]–[25]. We therefore examined the impact of TAM67 on AP1 factor interaction at the AP1-5 site. **Fig. 6** shows gel mobility shift analysis of AP1 factor binding to the hINV promoter AP1-5 site. **Fig. 6A** shows that the presence of TAM67-FLAG markedly increases the intensity of the gel shifted band (compare lanes 2 and 3) and that incubation with anti-FLAG produces a strong supershifted band only in cells expressing TAM67-FLAG (compare lanes 4 and 5). Moreover, the binding is competed by incubation with a 50-fold molar excess of radioinert AP1-5 oligonucleotide (see lanes 6 and 7), but a 50-fold excess of AP1-5 m does not compete (lane 8). We next examined the impact of TAM67 on endogenous AP1 factor interaction with AP1-5. As shown in **Fig. 6B**, supershifted bands (asterisks) are observed when extracts are incubated with anti-c-jun, junB, junD, Fra-1, Fra-2 and c-fos, and this interaction is reduced in the presence of TAM67-FLAG. Fos-B was not detected. The low signal intensity of the shifted bands is consistent with previous reports [47].

**Figure 6:** TAM67 binds to the AP1-5 site of hINV gene promoter. Keratinocytes were infected with 10 MOI tAd5-EV or tAd5-TAM67-FLAG and after 24 h nuclear extracts were prepared for gel shift. **A** TAM67 interaction with hINV promoter AP1-5 site. Nuclear extracts were incubated with AP1-5-P^32^ with or without a 50-fold molar excess of AP1-5 or AP1-5 m oligonucleotide, or anti-FLAG antibody, and electrophoresed on a 6% acrylamide non-denaturing gel. FP indicates free probe and NE is nuclear extract. The arrow indicates the major shifted bands and asterisks indicate supershifted bands. AP1-5 is an oligonucleotide encoding the AP1-5 site of hINV promoter. AP1-5 m is an AP1-5 mutant that does not bind AP1 transcription factors [47]. **B** TAM67 inhibits AP1 factor interaction with AP1-5. Nuclear extracts were incubated with AP1-5-P^32^ in the absence or presence of c-jun, junB, junD, Fra-1, Fra-2, c-fos, or fosB specific antibodies, and electrophoresed on a 6% acrylamide non-denaturing gel. Arrows indicate major shifted band and asterisks indicate supershifted bands. FP is free probe. **C** ChIP analysis reveals TAM67 presence at the hINV upstream regulatory region AP1-5 site *in vivo*. Nuclear extracts were prepared for ChIP analysis and incubated with anti-IgG or anti-FLAG and the precipitated DNA was analyzed for AP1-5 site encoding sequences. The values are mean ± SD (n = 3, p<0.001) and the asterisk indicates a significant increase compared to all other groups. Nucleotides −2218/−2055 encodes the AP1-5 site and nucleotides −1040/−919 is a region of the hINV upstream regulatory region that lacks an AP1 site.

To further assess the *in vivo* impact of TAM67 we used chromatin immunoprecipitation. Nuclear extracts from TAM67-FLAG positive and negative keratinocytes were prepared for ChIP analysis using a primer set that targets the AP1-5 binding site (−2218/−2005) and a second primer set that targets a region of the promoter lacking an AP1 factor binding site (−1040/−919). TAM67-FLAG and associated chromatin was precipitated with anti-FLAG. **Fig. 6C** shows that TAM67-FLAG is substantially enriched at the AP1-5 binding site (nucleotides −2218/−2055) as compared to the control DNA segment that lacks an AP1 binding site (nucleotides −1040/−919), suggesting TAM67 interaction at the hINV promoter AP1-5 site *in vivo*.

### TAM67 Impact on AP1 Factors *in vivo*

We previously described TAM67-rTA mice in which TAM67-FLAG expression can be induced in the suprabasal epidermis by addition of doxycycline to the drinking water [35]. Expression of TAM67 in this tissue would be expected to reduce expression of AP1 factor-regulated genes. To assess this, we compared expression of two AP1-factor regulated genes, involucrin and loricrin [10], [52], [53]. TAM67-rTA mice were treated for three days with doxycycline and total epidermal extracts were prepared to detect involucrin and loricrin. Consistent with the finding that involucrin expression is reduced in TAM67-expressing cultured keratinocytes, we find that involucrin level is reduced in TAM67 expressing mouse epidermis (**Fig. 7A**). We also show that loricrin protein level is reduced. Loricrin expression is also AP1 factor signaling dependent [52].

**Figure 7:** Impact of TAM67 on AP1 factors in vivo. TAM67-rTA mice were treated with (+) or without (−) 2 mg/ml doxycycline in drinking water for 3 days. **A** Murine epidermis was collected free of the dermis by high temperature separation as previously described [35]. Total extract was prepared for immunoblot to detect the indicated proteins. TAM67-FLAG was detected with anti-FLAG. **B** Interaction of TAM67 with AP1 site consensus element. Nuclear extracts were prepared from epidermis and incubated with AP1c-P^32^ and other probes as indicated. FP indicates free probe, NE indicates nuclear extract. Similar results were observed in each of three experiments. **C** Impact of TAM67 on interaction of endogenous AP1 factors with AP1 site element. Nuclear extracts were prepared from TAM67-negative and TAM67-expressing epidermis and incubated with the AP1c-P^32^ and antibodies as indicated. The complexes were then separated on a non-denaturing 6% polyacrylamide gel. FP indicates free probe and NE is nuclear extract. Note the reduction in jun factor binding in the presence of TAM67-FLAG (left panel). We did not observe a significant reduction in fos factor interaction in the presence of TAM67 (right panel).

We next examined the impact of TAM67 on endogenous AP1 factor DNA binding in mouse epidermis nuclear extracts. **Fig. 7B** shows an increase in the quantity of shifted AP1c-P^32^ probe in extract prepared from TAM67-expressing epidermis. This binding is specifically reduced by addition of excess radioinert AP1c, but is not competed by Sp1 consensus sequence. Moreover, TAM67-FLAG binding to AP1c-P^32^ is confirmed by anti-FLAG supershift (**Fig. 7B**). We also examined the impact of TAM67 on endogenous AP1 factor binding to DNA. The supershift analysis in **Fig. 7C** shows that TAM67 binding to the AP1 consensus element reduces c-jun, junB and junD interaction, with a strong reduction observed for junD. In contrast, Fra-2 and c-fos interaction is not altered by TAM67 and interaction of Fra-1 and FosB is below the limits of detection.

## Discussion

We recently expressed dominant-negative c-jun in murine epidermis and observed significant changes in epidermal phenotype [35]. These changes included increased cell proliferation, delayed differentiation and reduced tumor formation [35]. We presume that TAM67 is impacting AP1 target genes in this tissue and so in the present study we examine the TAM67 mechanism of action in more detail. We studied the role of dominant-negative c-jun (TAM67) in human epidermal keratinocytes and in an *in vivo* murine keratinocyte model of differentiation.

In cultured human keratinocytes TAM67-FLAG was detected in punctate foci in the center of the nucleus. Expression of TAM67 produced profound changes in AP1 transcription factor function. The first change we observed was a reduction in c-jun, junB and junD protein and mRNA level. The decrease in mRNA encoding the jun factors could be due to a reduction in mRNA stability or to a reduction in transcription. Further study with the c-jun promoter upstream regulatory region revealed a TAM67-dependent reduction in promoter activity. This reduction required the presence of AP1 transcription factor binding sites within the c-jun promoter. These findings are consistent with previous reports indicating that AP1 factor auto-regulate via a feedback loop [48], [54]–[57]. Our findings suggest that TAM67 binds to these elements, displacing other AP1 factors, and thereby suppresses c-jun transcription. In contrast, it is interesting that level of the fos family members (Fra-1, Fra-2 and c-fos) is not altered by TAM67. The loss of jun factors is also reflected in co-precipitation experiments. Fra-1, Fra-2 and c-fos co-precipitate with TAM67-FLAG, but junB and junD do not. Presumably, the reduction in junB and junD co-precipitation is due to reduced expression of these proteins. Surprisingly, c-jun, which is markedly reduced in level, does co-precipitate with TAM67. Perhaps c-jun homodimer formation is favored and TAM67, which retains the leucine zipper domain required for dimerization [26], may seek out and interact with residual c-jun in the cells.

An interesting finding is that the population of jun family transcription factors is highly depleted in TAM67-positive keratinocytes. This feature has not been previously appreciated. Since AP1 factor signaling requires jun family members as dimerization partners for jun and fos, the absence of jun factors is expected to severely limit AP1 factor signaling. An equally interesting feature is that expression of fos family members is not reduced. This suggests that fos family proteins are not regulated by an AP1 factor-dependent feedback loop in this system.

Second, we examined the impact of TAM67 on AP1 factor interaction with DNA. DNA gel shift experiments indicate that TAM67-FLAG interacts with the AP1 consensus DNA sequence, and that TAM67, at the level we achieve in these experiments, substantially reduces interaction of endogenous AP1 factors with DNA binding sites. Previous studies suggest that TAM67 forms transcriptionally inactive heterodimers with jun and fos family members [26]. These factors bind to the promoter of target genes, but are not able to activate transcription. This mechanism, called transcriptional quenching, leads to reduced target gene expression [26]. Our findings also suggest an additional mechanism. Protein-protein crosslinking and gel shift experiments strongly suggest that TAM67-FLAG homodimers are preferentially formed in these cells, and we suspect that this homodimer is a major AP1 factor complex that interacts with DNA. This would suggest that a major mechanism whereby TAM67 inhibits AP1 target gene expression in keratinocytes is TAM67 homodimer interaction with DNA to block endogenous AP1 factor access to these sites. It is also clear, as reported previously [26], that TAM67 forms heterodimers with jun and fos proteins, to form inactive complexes that quench activity of the complex. Thus, two mechanisms are possible: a blocking action wherein the TAM67 homodimer binds to DNA to block endogenous AP1 factor interaction with AP1 sites, and a quenching action wherein TAM67 inhibits the transactivation potential of endogenous AP1 factors by forming inhibitory TAM67:jun and TAM67:fos heterodimers (**Fig. 8**). Our studies favor the blocking mechanism involving TAM67 homodimers.

**Figure 8:** Mechanism of TAM67 action in keratinocytes. **A** Wild-type regulation involves the binding of fos:jun heterodimers (and jun:jun hetero and homodimers, not shown) to AP1 response element to drive differentiation-associated gene expression. Blocking occurs when the concentration of TAM67 present in the cells is high enough that TAM67 homodimers comprise the major complex bound to DNA and this complex blocks interaction of endogenous AP1 factors with the element. Quenching occurs when TAM67 complexes with endogenous jun and fos factors and this complex, which is transcriptionally inactive, binds to DNA. We propose that blocking is a major mechanism of TAM67 action in our system, but that quenching is also important. **B** TAM67 interaction at the promoter elements leads to blocking and quenching to reduce AP1 factor interaction and activity at AP1 binding sites. This leads to reduced expression of jun factors and ultimately reduced target gene (involucrin, loricrin) expression.

In addition, we examined the impact of TAM67 on an important AP1 transcription factor-regulated target, involucrin. Involucrin is a marker of suprabasal differentiation in epidermis that is regulated by a MAP kinase cascade [36], [47]. Activation of this cascade leads to AP1 factor interaction with specific DNA binding elements on the hINV promoter to drive expression [23]–[25]. A key DNA binding site that is required for involucrin expression, both in cultured keratinocytes and *in vivo*, is the AP1-5 DNA binding site located in the distal regulatory region of the hINV gene promoter [36], [47], [50]. We show that TAM67 reduces hINV mRNA and protein level in cultured keratinocytes. Moreover, hINV promoter activity is also reduced, suggesting that TAM67 is inhibiting AP1 factor-dependent transcription. We confirmed TAM67 interaction with AP1-5 transcription factor binding site in the hINV promoter by gel mobility shift and chromatin IP. These findings confirm the important role of the AP1-5 binding site in driving hINV gene expression [22]–[25]. The fact that this is associated with reduced binding of AP1 factor at this site, as measured by gel mobility supershift assay, suggests that TAM67 is displacing these factors by competition.

We also examined the impact of TAM67 expression on involucrin protein level in TAM67-expressing murine epidermis. We compared control mice (lacking TAM67 expression) and TAM67-expressing mice. These studies reveal a substantial reduction in murine involucrin protein in TAM67-expressing epidermis. This is associated with a 2 to 3-fold increase in transcription factor binding to the AP1 site in extracts prepared from TAM67-expressing epidermis. This increase is directly associated with increased TAM67 level, suggesting that TAM67 is a major factor interacting with the AP1 binding elements in the epidermis of these mice. TAM67 appears to readily compete jun family factors off from this site, but appears less efficient at competing fos family factors. We suspect that this is due preferred interaction with jun factors and to the somewhat lower level of TAM67 expression in mouse epidermis as compared to cultured keratinocytes.

In summary, we describe several findings regarding the mechanism of TAM67 action in keratinocytes and in TAM67-expressing murine epidermis. First, our findings suggest that AP1 transcription factors regulate c-jun, junB, junD mRNA and protein level. Moreover, we show that TAM67 inhibits activity of the c-jun promoter, suggesting a transcriptional mechanism of regulation. Second, we show that blocking AP1 factor access to the hINV gene promoter AP1 factor binding site inhibits transcription, both in cultured human cells and *in vivo* in mouse epidermis. Third, this inhibition appears to be mediated by a “blocking” mechanism where a TAM67 homodimer interacts with the AP1 response element to suppress transcription by preventing endogenous jun and fos factor binding to the element (**Fig. 8**). Crosslinking experiments suggest the presence of TAM67 homodimers as the major species present in keratinocytes. We suspect that the balance of TAM67 homodimers versus TAM67 heterodimerzation with endogenous jun and fos factors is depend upon the concentration of TAM67 expressed. At higher concentrations we would expect TAM67 homodimers to be the major species and that these factors will block endogenous AP1 factor interaction with DNA. An alternate mechanism, quenching, where TAM67 forms heterodimers with fos and jun proteins to produce a transcriptionally inactivate complex at AP1 DNA binding sites, is also likely. Crosslinking and co-immunoprecipitation experiments suggest some formation of TAM67 heterodimers with endogenous AP1 factors. An additional mechanism, called squelching (not shown), is also possible [26], [58], [59]. In this mechanism an inhibitor protein interacts with endogenous factors involved in transcription regulation that are not bound to DNA [26], [58], [59]. Although this may also be a mechanism of TAM67 inhibition, wherein TAM67 sequesters co-activator proteins away from the AP1 binding sites, we suspect that the major mechanisms whereby TAM67 suppresses gene expression in keratinocytes are AP1 site blocking and quenching (**Fig. 8A**) leading to suppression of jun factor and target gene (hINV, loricrin) expression (**Fig. 8B**). Our results suggest that these mechanisms are active both in cultures keratinocytes and in TAM67-expressing murine epidermis.

## Materials and Methods

### Cell Culture and Virus Infection

Primary cultures of human newborn foreskin keratinocytes were cultured in keratinocyte serum-free medium (KSFM) supplemented with epidermal growth factor and bovine pituitary extract (10724, Gibco, Invitrogen, Carlsbad, CA). These are obtained as discarded tissue samples and their use was reviewed and approved in writing by the University of Maryland Human Subjects Institutional Review Board. For virus infection, cells were plated at 40% confluence (0.5 million cells per 21 cm^2^ dish) and infected with 0, 2 or 10 MOI of tAd5-EV or tAd5-TAM67-FLAG in the presence of 5 MOI of Ad5-TA virus in KSFM containing 6 µg/ml polybrene (H9268, Sigma, St. Louis, MO). After 6 h the cells were washed and shifted to fresh virus-free medium.

### Immunological Methods and Antibodies

For immunoblot, keratinocytes were washed twice with phosphate-buffered saline (PBS), drained, and 0.5 ml of lysis buffer (20 mM Tris-HCl, pH 7.5, 150 mM NaCl, 1 mM Na_2_EDTA, 1 mM EGTA, 1% Triton X-100, 2.5 mM sodium pyrophosphate, 1 mM β-glycerophosphate, 1 mM Na_3_VO_4_ and 1 µg/ml leupeptin) supplemented with protease inhibitors was added to each 21 cm^2^ (60 mm) dish. After 5 min on ice, the cells were collected by scraping, and pelleted and sonicated. After centrifugation at 4°C and 15,000×g for 10 min, protein aliquots containing 30 µg of protein were separated on denaturing and reducing Laemmli [60] 8% polyacrylamide gels and transferred to nitrocellulose. The membrane was blocked in PBS containing 5% milk powder and 0.1% Tween 20, and incubated at 4°C overnight with primary antibody and for 1 h at 25°C with horseradish peroxidase-conjugated secondary antibody. Antibody binding was visualized using chemiluminescence detection reagent [61].

For anti-FLAG immunoprecipitation, keratinocytes were infected with 10 MOI of tAd5-EV or tAd5-TAM67-FLAG with 10 MOI of Ad5-TA. At 24 h, 200 µg of total cell extract was diluted to final volume of 500 µl in lysis buffer and pre-cleared by addition of 25 µl of protein A/G-agarose for 1 h at 4°C. The samples were then incubated with 20 µl of anti-FLAG M2 affinity gel (Sigma, A2220) overnight, and the antibody complex was washed three times with lysis buffer and boiled in 40 µl of Laemmli sample buffer for electrophoresis.

### Immunofluorescence

Keratinocytes, growing on coverslips, were rinsed with PBS and fixed with 1∶1 acetone:methanol for 10 min at −20°C. Cells were washed three times in PBS for 5 min, and the coverslips were blocked in 3% bovine serum albumin in PBS for 1 h at room temperature and then incubated with monoclonal anti-FLAG M2 antibody (F3165, Sigma, diluted 1∶1000) for 1 h at room temperature. Coverslips were washed three times in PBS for 5 min each and incubated with Alexa Fluor 488-conjugated goat anti-mouse IgG (A11029, Invitrogen, Eugene, OR, diluted 1∶1000) for 45 min at room temperature. Cells were further co-stained with 2 µg/ml Hoechst 33258 (H3569, Invitrogen) for 5 min, rinsed in PBS and place in mounting medium (M1289, Sigma). Fluorescence was visualized using an Olympus OX81 spinning-disc confocal microscope. No signaling was detected in the absence of primary antibody.

### Antibodies

Rabbit polyclonal antibodies including anti-c-jun (sc-1694, diluted 1∶1000), anti-jun D (sc-74×, diluted 1∶500), anti-Fra-1 (sc-605×, diluted 1∶1000) and anti-Fra-2 (sc-604×, diluted 1∶1000), and mouse anti-junB (sc-8051, diluted 1∶300) and goat anti-fosB (sc-482, diluted 1∶300) were obtained from Santa Cruz Biotechnology (Santa Cruz, CA). Rabbit polyclonal anti-c-fos (ab7963, diluted 1∶500) was from Abcam (Cambridge, UK). Monoclonal anti-FLAG M2-Peroxidase (A8952, diluted 1∶3000) and monoclonal anti-β-Actin (A1978, diluted 1∶3000) were purchased from Sigma (St. Louis, MO). Rabbit anti-human involucrin (hINV) serum (diluted 1∶2000) was produced in our laboratory [62]. Donkey anti-rabbit (NA934, diluted 1∶3000) and sheep anti-mouse HRP-conjugated secondary antibody (NA931, diluted 1∶3000) were from GE Healthcare (GE Healthcare, Piscataway, NJ). Donkey anti-goat HRP-conjugated secondary antibody (sc-2033, diluted 1∶3000) was from Santa Cruz Biotechnology (Santa Cruz, CA). Rabbit anti-loricrin (PRB-145P, diluted 1∶1000) was obtained from Covance (Princeton, NJ).

### Nuclear Extract Preparation

Keratinocytes (5×10^6^ cells) were harvested with trypsin-EDTA, collected by centrifugation at 500×g and washed several times with PBS. Nuclear pellet and cytoplasmic fractions were prepared using Nuclear and Cytoplasmic Extraction Kit (78833, Pierce Biotechnology, Rockford IL) and stored at −80°C. For protein crosslinking, the pellet (nuclear fraction, 5×10^6^ cell equivalents) was suspended in 100 µl of PBS (pH 8.0) containing 1 mM disuccinimidyl suberate (DSS, 21555, Pierce, Rockford, IL) and incubated for 10 min at room temperature. Tris-HCl (1 M, pH 7) was added to a final concentration of 10 mM to stop the reaction, and the protein samples were used for gel electrophoresis and immunoblot.

To prepare nuclear extract from mouse epidermis, skin was removed and placed on ice and the epidermis was removed by scraping with a razor blade. Nuclear extract was prepared from the epidermal tissue using the nuclear and cytoplasmic extraction kit (78833, Pierce Biotechnology, Rockford, IL) and stored at −80°C.

### Chromatin Immunoprecipitation Assay (ChIP)

ChIP assay was performed as described [63] with minor modification. Keratinocytes (5×10^5^ cells) from a 35 mm dish were crosslinked with 1.42% formaldehyde at room temperature for 15 min followed by quenching with 125 mM glycine and then washed with ice cold PBS containing histone deacetylase inhibitors. The cells were then lysed in 150 µl of lysis buffer (50 mM Tris-HCl, pH 8, 10 mM EDTA, 1% SDS, 1 mM PMSF, 20 mM sodium butyrate, and protease inhibitors). Samples were chilled on ice and DNA was sheared using a Branson Sonifier (three 30-sec pulses on ice at 40% amplitude with 30 seconds between pulses to produce fragments of 1,000 bp). Four hundred microliters of RIPA buffer containing protease inhibitors and histone deacetylase inhibitors was added followed by a centrifugation of 12,000×g for 10 min. Aliquots of supernatant containing sheared chromatin were used for immunoprecipitation. Mouse monoclonal anti-FLAG (2 µg, F3165, Sigma, St. Louis, MO) was added to Dynabeads Protein A and incubated for 2 h at 4°C with rotation at 40 rpm. Sheared chromatin was added and mixture was incubated at 4°C overnight with rotation. The chromatin-antibody complex was washed twice with RIPA buffer and 40 µl of Chelex 100 slurry (10% wt/vol) was added to the washed beads prior to boiling for 10 min. The samples were then treated with proteinase K for 30 min at 55°C and boiled for 10 min. Enrichment of TAM67-FLAG-associated DNA sequences in immunoprecipitated samples and input samples were detected by quantitative RT-PCR using sequence specific primers and LightCycler 480 SYBR Green I Master mix. ChIP primers included hINV promoter AP1-5 (nucleotides −2218/−2055) forward: 5′-TCAGCTGTATCCACTGCCCTCTTT-3′ and reverse: 5′-TCACACCGGTCTTATGGGTTAGCA-3′ primers, and hINV promoter control (nucleotides −1040/−919) forward: 5′-CCTCTCAGGGAGAGATTGACATGA-3′ and reverse: 5′-CAACAGTGCACCAGCACACTTGAA-3′ primers [23].

### Gel Mobility Shift Assays

Cells were washed with PBS for preparation of nuclear extract using NE-PER Nuclear and Cytoplasmic Extraction Reagent (78833, Pierce Biotechnology, Rockford, IL). Binding of transcription factors to double-stranded AP1 consensus (AP1c) oligonucleotide 5′-CGCTTG**ATGAGTCAGC**CGGAA-3′ (E320A, Promega, Madison, WI, AP1 site in bold) or hINV AP1-5 probe which encodes the AP1-5 binding site in upstream regulatory region of human involucrin promoter, 5′-CTTAAGGCTCTTATTATGCCG**TGAGTCAG**AGGGCGGGAGGCAGATCT-3′ (AP1 site in bold, Sp1 site underlined) [50], was monitored by gel mobility shift assay. Three micrograms of nuclear extract was incubated for 30 min at room temperature in a volume of 20 µl containing 20 mM HEPES, pH 7.5, 10% glycerol, 50 mM KCl, 2 mM MgCl_2_, 0.5 mM EDTA, 0.5 mM DTT, 1 µg/ml poly(dI:dC), 0.1 mg/ml bovine serum albumin, and 40,000 cpm radioactive double-stranded AP1c-P^32^ or AP1-5-P^32^ oligonucleotide. For competition studies, a fixed molar excess of non-radioactive competitor oligonucleotide was added to the DNA binding reaction. These competitors included Sp1 consensus oligonucleotide (Sp1c) 5′-ATTCGATCGGGGCGGGGCGAGC-3′ (E323, Promega, Madison, WI, Sp1 site underlined), AP1c and AP1-5 m/Sp1 m, 5′-CTTAAGGCTCTTATTATGCCG**TGAGCCAG**AGTCA AGGAGGCAGATCT-3′ (AP1 site in bold, Sp1 site underlined, mutant nucleotides shaded) [50]. For gel mobility supershift assay, 2 µg of antibody specific for FLAG (F3165, Sigma, St. Louis, MO) or c-jun (sc-45×), junB (sc-46×), junD (sc-74×), Fra1 (sc-605×), Fra-2 (sc-604×), c-fos (sc-253×) and fosB (sc-48×) was added to the reaction mixture and incubated 1 h at 25°C. The ^32^P-labeled probe was then added and the incubation was continued for an additional 30 min at 25°C. Protein-DNA complexes were resolved in 6% polyacrylamide gels under nondenaturing conditions [8], [61].

### Quantitative RT-PCR

Total RNA was extracted using Illustra RNAspin Mini Isolation kit (25-0500-70, GE Healthcare) according to instructions. One microgram of total RNA was reverse-transcribed to cDNA using Superscript III reverse transcriptase (18080-093, Invitrogen Inc.) and random primers (10814270001, Roche, Indianapolis, IN). Gene expression was measured by quantitative PCR using Roche LightCycler 480 System and SYBR Green reagents (LightCycler 480 SYBR Green I Master, 04 707 516 001, Roche). RNA level was normalized to glyceraldehyde-3-phosphate dehydrogenase (GAPDH) mRNA level. Relative mRNA level was analyzed by the comparative C_T_ method. The primers, designed to detect the indicated genes in mRNA isolated from human keratinocytes, include (forward/reverse) glyceraldehyde-3-phosphate dehydrogenase 5′-TCCACTGGCGTCTTCACC-3′/5′-GGCAGAGATGATGACCCTTT-3′; c-fos 5′-TGTCTGTGGCTTCCCTTGATCTGA-3′/5′-TGGATGATGCTGGGAACAGGAAGT-3′; Fra-1 5′-CTGTGCTTGAACCTGAGGCA-3′/5′-GGTGAAAGGAGTTAGGGAGGGT-3′ [64]; Fra-2 5′-CCCTGCACACCCCCATCGTG-3′/5′-TGATTGGTCCCCGCTGCTACTGCTT-3′ [65]; c-jun 5′-GTACCTGATGAACCTGATGC-3′/5′-GGTCACAGCACATGCCACTT-3′ [66]; junB 5′-GTCACCGAGGAGCAGGAGG-3′/5′-TCTTGTGCAGATCGTCCAGG-3′ [66]; junD 5′-AAGACCCTCAAGAGTCAGAACACG-3′/5′-TGTTGACGTGGCTGAGGACTTTCT-3′; and involucrin 5′-CCTCAGCCTTACTGTGAG-3′/5′-GGGAGGCAGTGGAGTTGG-3′.

### hINV and c-jun Promoter Activity

Human involucrin hINV reporter plasmids, encoding various lengths of hINV promoter upstream regulatory region fused to the luciferase reporter gene have been described [36], [47]. We used hINV promoter constructs, pINV-2473, pINV-241, and pINV-41, which include nucleotides −2473/−7, −241/−7 and −41/−7, respectively, of the hINV promoter linked to the luciferase reporter gene [47]. TAM67 expression plasmid was pcDNA3-TAM67-FLAG. 12-O-Tetradecanoylphorbol-13-acetate (TPA) was obtained from Sigma (St. Louis, MO). For experiments, 2×10^5^ cells were seeded into 35 mm dishes 24 h before transfection. For transfection, 6 µl of Fugene-6 reagent (11 814 443 00, Roche, Indianapolis, IN) was mixed with 94 µl of KSFM, and incubated at 25°C for 10 min. This mixture was then added to 1 µg of hINV plasmid and 1 µg of TAM67-FLAG expression plasmid and incubated at 25°C for 20 min followed by direct addition to cultures containing 2 ml of KSFM. The final DNA concentration in all groups was maintained constant by addition of empty expression vector. At 24 h after transfection, 2 ml of fresh medium was added containing 0 or 50 ng/ml TPA. After an additional 24 h, the cells were washed with PBS and scraped into 200 µl of cell lysis buffer, and luciferase activity was assayed immediately. All assays were performed in triplicate, and each experiment was repeated a minimum of three times. Luciferase activity was normalized per microgram of protein. Promoter activity experiments were also performed in keratinocytes using c-jun promoter luciferase reporter constructs c-jun(−1780/+731) and c-jun(−1780/+731)-AP1 m which encode nucleotides −1780/+731 of the human c-jun promoter and upstream regulatory region [48]. The latter construct is identical except that the AP1 sites in the c-jun upstream regulatory region are mutated [48].

### TAM67-rTA Transgenic Mice

The TAM67-rTA mice are maintained in the genetic background as previously described [35]. These mice harbor a transgene that encodes TAM67-FLAG linked to a tetracycline-inducible promoter. Epidermis-specific TAM67-FLAG expression is induced by addition of 2 mg/ml doxycycline in drinking water and expression is maximal within two day [35]. A FLAG epitope is included at the carboxyl terminus of TAM67 so that expression can be easily monitored. For the experiments outlined in the present study we utilize 20 wk old female mice from TAM67-44 strain [35]. Epidermal extracts were prepared for gel mobility shift or immunoblot after a three day treatment with doxycycline. Mice were maintained in the University of Maryland School of Medicine animal facility in compliance with NIH regulations with laboratory chow and water accessible *ad libitum*. The study was approved by the University of Maryland School of Medicine Institutional Animal Care and Use Committee.
